RETRACTED

# Application Value of Color Doppler Ultrasonography Combined with Thyroid Autoantibody Tests in Early Diagnosis of Thyroid Cancer

**DOI:** 10.1155/2022/5248230

**Published:** 2022-04-27

**Authors:** Danlin Song, Fajin Dong, Jing Zheng, Hui Luo, Jinxi Wei

**Affiliations:** ^1^Department of Ultrasound, Shenzhen People's Hospital, 2nd Clinical Medical College of Jinan University, 1st Affiliated Hospital of Southern University of Science and Technology, Shenzhen, 518020 Guangdong, China; ^2^Department of Radiology, Shenzhen People's Hospital, 2nd Clinical Medical College of Jinan University, 1st Affiliated Hospital of Southern University of Science and Technology, Shenzhen, 518020 Guangdong, China

## Abstract

**Objective:**

To explore the application value of color Doppler ultrasonography combined with thyroid autoantibody tests in the early diagnosis of thyroid cancer.

**Methods:**

The medical data of 100 patients with thyroid nodules treated in our hospital from June 2019 to June 2021 were retrospectively analyzed; all patients received color Doppler ultrasonography and thyroid autoantibody tests before surgery and were divided into the benign lesion group (*n* = 45) and the malignant lesion group (*n* = 55) according to the postoperative pathological findings (the gold standard), so as to compare and analyze the application value of color Doppler ultrasonography, thyroid autoantibody tests, and their combination in the early diagnosis of thyroid cancer.

**Results:**

Compared with the pathological findings, the accuracy rate, sensitivity, specificity, positive predictive value, and negative predictive value of the combined diagnosis were significantly higher than those in the single diagnosis of color Doppler ultrasonography, TgAb test, TPOAb test, and TRAb test (*P* < 0.05), and by plotting the ROC curves to analyze the effect of these modalities in diagnosing early thyroid diseases, the results showed that the areas under the curve from large to small were combined diagnosis, color Doppler ultrasonography, TgAb test, TPOAb test, and TRAb test.

**Conclusion:**

Color Doppler ultrasonography has many advantages in the diagnosis of thyroid nodules, such as easy operation, painlessness, noninvasiveness, high efficiency, and repeatable detection, and the high-definition probe is able to show tiny lesions, echogenicity, blood flow signal, and other characteristics of foci. Combining color Doppler ultrasonography with testing thyroid autoantibodies such as TgAb, TPOAb, and TRAb can effectively improve the detection rate of early thyroid cancer, presenting significant reference value and meaning to clinical diagnosis and treatment of thyroid cancer.

RETRACTED

## 1. Introduction

Thyroid nodules are thyroid diseases with a high incidence rate in the clinic, which generally include benign thyroid nodules (nodular goiter, simple goiter, thyroid adenomas, etc.) and malignant thyroid nodules (thyroid cancer). Thyroid cancer is one of the more common malignant tumors in humans without obvious early symptoms, so early detection and treatment have very important clinical implications for the prognosis of cancer patients, and accurate early diagnosis strategies are crucial for the treatment and prognosis of thyroid cancer patients [1–4]. Although ultrasonography is the most commonly used and preferred imaging method for diagnosing thyroid in clinic with unique advantages, especially for early diagnosis, rational evaluation, precise staging, and timely treatment of thyroid gland, it has some limitations in terms of the visualization of tiny occult foci. Currently, research on early diagnosis of cancer is no longer limited to a certain kind of diagnostic modalities, and integrating multiple dimensions to look for efficient and practicable diagnostic strategies is a major research trend in the field. It is known from previous studies [5–7] that thyroid peroxidase antibody (TPOAb), thyroid-stimulating hormone receptor antibody (TRAb), and thyroglobulin antibody (TgAb) are all autoimmune thyroid disease-related autoantibodies as well as important indicators of studies on the risk factors for thyroid cancer, but some study conclusions [8] also argued that there is no direct evidence showing an association between them. Within such context, the clinical data of 100 patients with thyroid nodules treated in our hospital were retrospectively analyzed to explore the application value of combining color Doppler ultrasonography with thyroid autoantibody tests in the early diagnosis of thyroid cancer. The major contributions are the following: (1) The study improves the early diagnosis efficacy of thyroid cancer, increases the clinical concern in patients with low-risk thyroid cancer, and guides clinical treatment to reserve the gland function of such patients to the greatest extent and avoid unnecessary diagnosis and treatment. (2) Currently, the determination of benignancy and malignancy of thyroid nodules is still the important means for early diagnosis of thyroid cancer, and ultrasound, which is easy to operate and promote, is a good choice for initial screening, and jointly applying ultrasound with the thyroid autoantibody test can improve the early diagnostic efficacy of thyroid cancer.

## 2. Material and Methods

### 2.1. Case Screening and Grouping

The following are the inclusion criteria: (1) the patients were diagnosed with a benign thyroid nodule or thyroid cancer according to the postoperative pathological findings; (2) the patients met the surgical indications; (3) the patients did not receive any intervention treatments before surgery; (4) the patients received color Doppler ultrasonography and thyroid autoantibody tests; (5) the patients had complete clinical data, and the patients and their family members made an informed decision to join the review and analysis of the patients' clinical data for this study; and (6) the patients were diagnosed for the first time in our hospital. The following are the exclusion criteria for the patients: (1) complicated with hyperthyroidism, Hashimoto thyroiditis, etc.; (2) complicated with autoimmune dysfunction or coagulation disorders; (3) presence of history of thyroid surgery or treatment; (4) presence of cognitive disorder, common language disorder or seeing-hearing disorder, etc.; (5) pregnant or lactating women; and (6) low compliance and refused to accept subsequent follow-up. According to the statistical problems corresponding to the study objective and referring to the formula [9], relevant parameters were determined, and by combining with various limitations of the study, the finally determined number of sample cases was 100. Then, the medical data of 100 patients with thyroid nodules treated in our hospital from June 2019 to June 2021 were screened out, and all patients were divided into the benign lesion group (*n* = 45) and malignant lesion group (*n* = 55) according to their postoperative pathological findings. The study met the World Medical Association Declaration of Helsinki (2013) [10].

RETRACTED

### 2.2. Color Doppler Ultrasonography

The patients were in the supine position with their necks exposed, the color Doppler ultrasonic diagnostic apparatus (model: HD15; manufacturer: PHILIPS company) was used, with the probe frequency of 10.0 MHz. First, two-dimensional ultrasound was performed to observe the position, size, morphology, internal echogenicity, etc., of the thyroid and the number, size, and morphology of intraglandular masses and at the same time closely monitor the mass for encapsulation, posterior failure, and lymphadenectasis, with particular attention paid to echogenic foci [11–13]. Then, the color Doppler flow imaging instrument was used to further observe the thyroid mass for internal status and peripheral blood flow change and record the relevant parameters in detail.

### 2.3. Thyroid Autoantibody Tests

After 12 h of fasting, the proper amount of venous blood was drawn from all patients for thyroid autoantibody tests. The automatic electrochemiluminescence instrument (model: Roche Cobas 601; manufacturer: F. Hoffmann-La Roche Ltd.) was used to measure the level of TPOAb and TRAb, and the human anti-TgAb enzyme-linked immunoassay was applied to measure the TgAb level. Relevant detection kits were purchased from Wuhan Easy Diagnosis Biomedicine Co., Ltd.

RETRACTED

### 2.4. Evaluation Standards

If TgAb > 60 U/ml, TPOAb > 60 U/ml, or TRAb > 1.75 IU/L, it was determined that the diagnostic result was positive; when combining color Doppler ultrasonography with thyroid autoantibody tests, if one of the results showed positive, it was regarded as positive, and the postoperative pathological findings were considered the gold standard.

### 2.5. Statistical Processing

In this study, the between-group differences of data were calculated by SPSS22.0, the picture drawing software was GraphPad Prism 7 (GraphPad Software, San Diego, USA), the items included were enumeration data and measurement data, which were, respectively, expressed by [*n*(%)] and $\left(\bar{x}\pm s\right)$ and examined by *χ*^2^ test and *t*-test, and differences were considered statistically significant at *P* < 0.05.

## 3. Results and Analysis

### 3.1. General Data

No statistical differences in patients' general data such as age, BMI, diameter of nodule, gender, educational degree, and TNM stage between the two groups were observed (*P* < 0.05) (see Table 1).

### 3.2. Comparative Analysis with Pathological Findings

Compared with the pathological findings, the accuracy rate, sensitivity, specificity, positive predictive value (PPV), and negative predictive value (NPV) of the combined diagnosis were significantly higher than those in the single diagnosis of color Doppler ultrasonography, TgAb test, TPOAb test, and TRAb test (*P* < 0.05) (see Tables 2 and 3).

### 3.3. ROC Curve

By plotting the ROC curves to analyze the effect of these modalities in diagnosing early thyroid diseases, the results showed that the areas under the curve from large to small were combined diagnosis, color Doppler ultrasonography, TgAb test, TPOAb test, and TRAb test (see Figure 1 and Table 4).

## 4. Discussion

The thyroid gland, the largest and most important endocrine gland in the human body, is relatively accessible because of its superficial location and fewer variation in vascularity, which also provides good congenital conditions for ultrasonography. Color Doppler ultrasonography, with its advantages of easy operation, low cost, and high safety and accuracy, is considered to be the first choice for clinically diagnosing the nature of thyroid nodules and is often used in the preoperative diagnosis of thyroid cancer and the development of a surgical protocol [14–16]. The diagnosis and differentiation of thyroid cancer by color Doppler ultrasonography are mainly based on the two-dimensional morphological features and color Doppler flow status, which are generally reflected in the following aspects: (1) the morphology of the foci is irregular, and many of them are unifocal, accompanied by a spiculated margin; (2) the foci show heterogeneous echogenicity, uneven intensity, and attenuation posteriorly; (3) there are calcifications and abundant blood flow signals within the foci, which often show penetrating blood flow and relatively disorganized vascularity; and (4) pulsed Doppler shows that the flow in the feeding arteries appears as high velocity and hyperresistance, which may also be accompanied by a reverse flow spectrum in some patients [17–20]. Therefore, two-dimensional ultrasound can clearly observe the margin and the internal echogenicity of the foci, and on this basis, color Doppler ultrasonography can accurately monitor the vascularity and blood flow signal at the foci and make more accurate judgment on thyroid cancer, which indicates that color Doppler ultrasonography is feasible to diagnose thyroid cancer. The study also concluded that in diagnosing malignant and benign thyroid nodules, color Doppler ultrasonography obtained an accuracy rate of 89%, sensitivity of 90.74%, specificity of 86.96%, PPV of 89.09%, and NPV of 88.89%, and the area under the ROC curve reached up to 0.89, making it close to the pathological findings. The results were consistent with the report by Yang et al. [21], which further proved that color Doppler ultrasonography has higher diagnostic efficacy in early thyroid cancer and can serve as the first choice for diagnosing this disease.

RETRACTED

TRAbs are a heterogeneous class of specific immunoglobulins, which are divided into two subtypes, thyroid stimulating antibodies (TSAb) and thyroid blocking antibodies (TBAb); the former is associated with the pathogenesis of autoimmune hyperthyroidism (i.e., Grave's disease), and the latter is related to autoimmune hypothyroidism (mainly referred to as Hashimoto's disease). TgAb and TPOAb belong to specific thyroid autoantibodies, which are produced due to the damage of thyroid cells and leakage of cytosolic peroxidase (the key enzyme for the synthesis of thyroid hormone) and thyroglobulin into the blood stimulating body, and are likewise the marker antibodies of autoimmune thyroiditis. Their increased levels indicate that thyroid tissue is in an active state of immune inflammation, so both of them are the first indicators for the diagnosis of thyroid autoimmune diseases [22–25]. Compared with the pathological findings, the study results showed that the diagnostic efficacy of TgAb for benign and malignant thyroid lesions was higher than that of TPOAb and TRAb, but the diagnostic efficacy of all the single tests of these indicators was dissatisfied.

RETRACTED

In addition, compared with the pathological findings, the accuracy rate, sensitivity, specificity, PPV, and NPV of combining color Doppler ultrasonography with testing thyroid autoantibodies such as TgAb, TPOAb, and TRAb were significantly higher than those in the single diagnosis of color Doppler ultrasonography, TgAb test, TPOAb test, and TRAb test (*P* < 0.05), and by plotting the ROC curves to analyze the effect of these modalities in diagnosing early thyroid diseases, the results showed that the areas under the curve from large to small were combined diagnosis, color Doppler ultrasonography, TgAb test, TPOAb test, and TRAb test. The combined diagnosis obtained an accuracy rate of 93%, sensitivity of 94.44%, specificity of 94.45%, PPV of 92.73%, and NPV of 93.33%, and the area under the ROC curve reached up to 0.93, implying that combining color Doppler ultrasonography with testing thyroid autoantibodies including TgAb, TPOAb, and TRAb could significantly improve the early diagnostic efficacy of thyroid cancer. It is a retrospective analysis study, and patients' data and information are the key to guaranteeing the process of the study, which also will bring limitations, so this article did not provide an in-depth analysis of the malignancy of thyroid cancer patients, and exploration can be launched in this direction in subsequent studies.

## 5. Conclusion

In conclusion, color Doppler ultrasonography has many advantages in the diagnosis of thyroid nodules, such as easy operation, painlessness, noninvasiveness, high efficiency, and repeatable detection, and the high-definition probe is able to show tiny lesions, echogenicity, blood flow signal, and other characteristics of foci. Combining color Doppler ultrasonography with testing thyroid autoantibodies such as TgAb, TPOAb, and TRAb can effectively improve the detection rate of early thyroid cancer, presenting significant reference value and meaning to clinical diagnosis and treatment of thyroid cancer.

## Figures and Tables

**Figure 1:** ROC curves.

**Table 1:** General data.

Group	*n*	Age (years)	BMI (kg/m^2^)	Diameter of nodule (cm)	Gender (male/female)
Benign lesion group	45	48.15 ± 8.22	24.12 ± 3.07	2.96 ± 0.30	19/26
Malignant lesion group	55	47.86 ± 7.93	24.25 ± 3.03	2.94 ± 0.31	25/30
*χ* ^2^/*t*		0.179	0.212	0.326	0.105
*P*		0.858	0.832	0.745	0.746

**Table 2:** Results from color Doppler ultrasonography, TgAb test, TPOAb test, TRAb test, and pathological findings.

Pathological findings	*n*	Combined diagnosis		Color Doppler ultrasonography		TRAb		TPOAb		TgAb	
		+	−	+	−	+	−	+	−	+	−
+	55	51	3	49	5	46	9	45	11	43	12
−	45	4	42	6	40	9	36	10	34	12	33

RETRACTED

**Table 3:** Diagnosis efficacy of color Doppler ultrasonography, TgAb test, TPOAb test, and TRAb test.

Test variables	Accuracy rate	Sensitivity	Specificity	PPV	NPV
Combined diagnosis	93.00	94.44	95.45	92.73	93.33
Color Doppler ultrasonography	89.00^∗^	90.74^∗^	86.96^∗^	89.09^∗^	88.89^∗^
TgAb	82.00^∗^	83.64^∗^	80.00^∗^	83.64^∗^	80.00^∗^
TPOAb	79.00^∗^	80.36^∗^	77.27^∗^	81.82^∗^	75.56^∗^
TRAb	76.00^∗^	78.18^∗^	73.33^∗^	78.18^∗^	73.33^∗^

Note: ∗ denoted statistically significant difference versus combined diagnosis (*P* < 0.05).

**Table 4:** Area under curve.

Test result variable	Area	S.E.^a^	Sig.^b^	Asymp. 95% CI
Combined diagnosis	0.930	0.030	0.000	0.872-0.988
Color Doppler ultrasonography	0.890	0.037	0.000	0.818-0.961
TgAb	0.818	0.045	0.000	0.730-0.907
TPOAb	0.787	0.048	0.000	0.693-0.881
TRAb	0.758	0.050	0.000	0.659-0.856

Note: a denoted nonparametric hypothesis; b denoted null hypothesis: real area = 0.5; Sig was short for “significance”.

## Data Availability

Data to support the findings of this study is available on reasonable request from the corresponding author.
